The article "Observation and Nursing of Adverse Reactions in Severe Patients with Enhanced MRI" was retracted in 2023. Reasons: suspected computer-generated content; unreliable results or conclusions; concerns about the data; concerns about the results or conclusions.

# Observation and Nursing of Adverse Reactions in Severe Patients with Enhanced MRI

**DOI:** 10.1155/2022/5319179

**Published:** 2022-03-30

**Authors:** Yehua Dai, Changneng Peng, Pan Li

**Affiliations:** ^1^Nursing School, Xiangnan University, Chenzhou, China; ^2^No. 4 People's Hospital of Chenzhou City, Chenzhou, China

## Abstract

In order to explore the observation and nursing of adverse reactions in severe patients with enhanced magnetic resonance imaging, a family nursing service model was proposed in patients with enhanced magnetic resonance imaging. 150 patients who underwent enhanced magnetic resonance imaging in a hospital were selected as the research objects. The patients were divided into two groups by random number table method. 75 patients in the control group received routine nursing intervention and 75 patients in the observation group received family nursing service intervention. The anxiety score, depression score, examination time, one-time success rate, comfort score, incidence of adverse reactions, excellent image quality rate and nursing satisfaction were compared between the two groups. The results showed that the anxiety score and depression score of the observation group were lower than those of the control group (*P* < 0.05), the examination time of the observation group was significantly shorter than that of the control group (*P* < 0.05), and the comfort score and one-time success rate of the observation group were significantly higher than those of the control group (*P* < 0.05). The incidence of adverse reactions was significantly lower than that in the control group (*P* < 0.05), the excellent and good image quality rate (95.00%) and nursing satisfaction (97.22%) were significantly higher than those in the control group (83.00%, 86.56%). This shows that the application effect of family nursing service mode in magnetic resonance enhanced scanning is remarkable. Therefore, the use of family care mode in MRI patient examination can effectively reduce patients' anxiety and depression scores, shorten examination time, reduce adverse reactions, improve the success rate of one-time examination, improve patients' comfort during examination and patients' evaluation of nursing services. The effect is ideal and worthy of clinical research and promotion.

## 1. Introduction

Magnetic resonance imaging technology is a medical examination technology that provides a reliable basis for the diagnosis of clinical diseases. Compared with the previous medical imaging technology, it has higher resolution for soft tissue, can display more lesions that cannot be displayed by CT, and identify the nature and scope of lesions. It has the advantages of accuracy, safety and reliability [1]. Magnetic resonance imaging (MRI) scan has many contraindications, long inspection time and high machine noise. The patient is in a passive position for a long time and is in a large instrument with narrow space. It is easy to produce negative emotions such as fear, irritability, depression and anxiety. Some patients can not complete the examination due to noise and body position discomfort, which reduces the patient's cooperation compliance and adversely affects the scanning results [2,3]. High quality nursing is that nurses integrate the nursing concept of “people-oriented and patient-centered” and humanistic care into nursing work, and provide high-quality nursing services for patients on the basis of basic nursing and routine nursing services [4,5].  Figure 1 is a technical scheme of an image reconstruction system and method in magnetic resonance imaging. The success of MRI scanning has a direct impact on the diagnosis of the disease. High quality nursing service is the key to ensure the successful and safe completion of MRI scanning and ensure the image quality [6,7]. Masuda, R. and others pointed out that effective nursing intervention for patients undergoing MRI Dynamic enhancement scanning can alleviate their negative emotions before the examination and maintain a peaceful state of mind during the examination, so as to help them successfully complete the examination [8]. Clinical research shows that effective nursing intervention for patients undergoing MRI Dynamic enhancement scanning can improve their negative emotions before examination and make them complete the examination smoothly.

The article "Observation and Nursing of Adverse Reactions in Severe Patients with Enhanced MRI" was retracted in 2023. Reasons: suspected computer-generated content; unreliable results or conclusions; concerns about the data; concerns about the results or conclusions.

Family nursing service mode is a new nursing mode, which can be applied to MRI examination. The nursing core of this nursing mode is “family affection”, that is, through nursing intervention, patients can feel family care. The purpose of this study was to explore the application effect of family nursing service mode in patients undergoing enhanced magnetic resonance imaging. Therefore, a single blind controlled study was conducted on 150 patients undergoing enhanced magnetic resonance imaging in our hospital. In the examination of patients with MRI, the family care mode can effectively reduce the scores of anxiety and depression, shorten the examination time, reduce adverse reactions, improve the success rate of one-time examination, improve the comfort of patients during examination, and improve the scores of patients on nursing services. The effect is ideal, which is worthy of clinical research and promotion.

## 2. Research Methods

### 2.1. Data and Methods

#### 2.1.1. General Information

150 patients who underwent enhanced magnetic resonance imaging in a hospital were selected as the research objects. All patients underwent enhanced magnetic resonance imaging (MRI), had no allergic reaction to the developing contrast agent, had informed consent to the study and participated voluntarily. This study was approved by the hospital ethics committee in advance. The patients were randomly divided into two groups. There were 75 cases in the control group, 39 males and 36 females. The age ranged from 23 to 59 years (40.81 ± 17.24 years). There were 75 patients in the observation group, 37 males and 38 females. The age ranged from 22 to 58 years (40.19 ± 16.83 years). There was no significant difference in age and gender between the two groups (*P* > 0.05).

The article "Observation and Nursing of Adverse Reactions in Severe Patients with Enhanced MRI" was retracted in 2023. Reasons: suspected computer-generated content; unreliable results or conclusions; concerns about the data; concerns about the results or conclusions.

### 2.2. Method

#### 2.2.1. Intervention Methods

Control group. 75 patients received routine nursing intervention, prepared for the examination before the examination, guided the patients how to place the correct body position during the examination, and observed and treated whether the patients had adverse reactions after the examination.

Observation group. 75 patients received the intervention of family nursing service mode, the basic nursing measures were the same as those in the control group, and the concept of “family nursing” was added to the nursing service, as follows. ① Before examination: explain the importance of MRI Dynamic Enhanced scanning to disease diagnosis for patients and their families in easy to understand language, inform patients of the cooperation points and relevant precautions of MRI enhanced scanning, communicate well with patients, and give family care to patients. ② During examination: during the examination, ensure that the indoor air quality is good and the temperature and humidity are appropriate, so as to improve the patient's comfortable experience as much as possible, and properly prepare blankets or quilts and other items to prevent cold and keep warm. ③ After examination: send the patient to the observation room, tell the patient to observe for at least 30 min, ask the patient's family members to accompany the patient, comfort the patient, and closely observe the patient. If there is no abnormality in the observation for 30 min, the observation can be ended [9].

#### 2.2.2. Observation Index

The anxiety score, depression score, examination time, one-time success rate, comfort score, incidence of adverse reactions, excellent image quality rate and nursing satisfaction were compared between the two groups. Among them, Anxiety score and depression score are respectively assessed by self rating Anxiety Scale (SAS) in Table 1 and self rating Depression Scale (SDS) in Table 2. The full score is 100. The higher the score, the more serious its negative psychology is; the comfort evaluation tool is comfort scale (General comfort questionnaire, GCQ), the score is 28 ∼ 112. The higher the score, the more comfortable it is. The image quality is divided into excellent, good and poor. Excellent means that the image is clear and free of artifacts. Good means that there are a small amount of artifacts but do not interfere with the diagnosis result. Poor means that there are many artifacts and interfere with the diagnosis result. Excellent rate = excellent rate + good rate. Nursing satisfaction is scored by patients, with a full score of 100, 80 ∼ 100 being very satisfied, 60 ∼ 79 being relatively satisfied, less than 60 being dissatisfied, satisfaction = (very satisfied + relatively satisfied) cases/total cases × 100％。

The article "Observation and Nursing of Adverse Reactions in Severe Patients with Enhanced MRI" was retracted in 2023. Reasons: suspected computer-generated content; unreliable results or conclusions; concerns about the data; concerns about the results or conclusions.

#### 2.2.3. Statistical Methods

The data were processed by spss19.0 software. The counting data were represented by [cases (%). *x*^2^ test was performed. The measurement data were represented by mean ± standard deviation $\left(\bar{x}\pm s\right)$. *T* test was performed. The difference was statistically significant with *P* < 0.05.

## 3. Result Analysis

### 3.1. Comparison of Anxiety and Depression Scores between the Two Groups

Comparison of anxiety, depression and comfort scores between the two groups after intervention: after intervention, the anxiety and depression scores of nursing objects in the experimental group were significantly lower than those in the control group, and the comfort scores were significantly higher than those in the control group (*P* < 0.05). See Table 3.

### 3.2. Comparison of Examination Time, Comfort, and Nursing Score between the Two Groups

The examination time of the observation group was significantly less than that of the control group, and the comfort score and nursing score of the observation group were significantly higher than those of the control group (*P* < 0.05), as shown in Table 4.

### 3.3. One Time Success Rate and Adverse Reaction Rate of the Two Groups

The one-time success rate in the observation group was 75%, higher than 68% in the control group. The number of adverse reactions was 4, lower than 13 in the control group. The difference was statistically significant (*P* < 0.05), as shown in Table 5.

### 3.4. Comparison of Inspection Quality between the Two Groups

The excellent rate of MRI, the success rate of one-time examination and the satisfaction rate of examination and nursing in the observation group were significantly higher than those in the control group (*P* < 0.05). See Table 6, Figure 2.

### 3.5. Comparison of Nursing Satisfaction Rate between the Two Groups

The total satisfaction rate of patients in the observation group was higher than that in the control group (*P* < 0.05). See Table 7 and Figure 3 for details.

The article "Observation and Nursing of Adverse Reactions in Severe Patients with Enhanced MRI" was retracted in 2023. Reasons: suspected computer-generated content; unreliable results or conclusions; concerns about the data; concerns about the results or conclusions.

## 4. Discussion

However, due to the need to inject contrast agent during MRI enhancement scanning, there may be adverse reactions during the examination. In addition, some patients have anxiety before the examination due to insufficient cognition of MRI enhancement scanning, which is unfavorable to the development of the examination. Therefore, nursing measures should also be taken to intervene in the process of nuclear MRI enhancement imaging [10,11].

Because patients have less awareness of the examination and are worried about the damage caused by radiation to the body, they think that the injection of contrast agent may have adverse reactions, cannot cooperate well, affect the smoothness, and even refuse not to cooperate [12]. Therefore, appropriate psychological counseling and its necessity, the hospital applied the family nursing model in the enhanced examination. When arranging patients' appointment for examination, priority should be given to acute and critical patients, old, weak, children and those who have a long way to go. Before the examination, communicate with the patient in easy to understand language, carefully explain the necessity and safety of the examination, equip the drugs, equipment and rescue supplies required for the examination, carefully answer the patient's questions, meet their reasonable requirements, and alleviate tension and fear. The waiting hall shall be kept clean and tidy, equipped with books and pictures, film and television broadcasting system, sufficient seats and drinking water equipment to facilitate patients to save valuables, equipped with a locked extraction cabinet, the room temperature shall be controlled at 18 ∼ 25°C, the humidity shall be 50% ∼ 60%, keep the room clean and quiet, and prepare blankets, sheets and examination clothes for patients to prevent catching cold [13,14]. Patients should be given family support during the examination to ensure that they use a comfortable position during the examination. Due to the narrow examination space and long examination time, patients can be instructed to close their eyes or wear eye masks to calm their tension, inform patients that the examination time is long and make them psychologically prepared. After the examination, the home belongs to the lounge to accompany the patient. For critically ill patients and critical values, the receiving doctor shall be informed to issue the examination report as soon as possible. For slow patients, the time and place of taking the report shall be informed, and a written description shall be given if necessary. When the patient lives far away or it is inconvenient for the patient to get the report, the report can be mailed by express, and the mailing address and basic information of the patient shall be recorded without confusion. It is strictly prohibited to discuss the patient's condition and patient privacy in front of the patient. For adverse diseases such as suspected malignant tumors, try to notify the family members to get the report and take protective medical measures [15,16].

The article "Observation and Nursing of Adverse Reactions in Severe Patients with Enhanced MRI" was retracted in 2023. Reasons: suspected computer-generated content; unreliable results or conclusions; concerns about the data; concerns about the results or conclusions.

In the tense nurse patient relationship in China, the great part that affects patients' satisfaction with nursing staff is nursing attitude. Due to medical conditions, most nursing staff are overloaded, and most of them have no energy to communicate with patients in one day's work. According to the scientific ratio of nursing staff to patients, the hospital provides professional nursing family training to narrow the relationship between nurses and patients and strengthen mutual intimacy and trust [17]. It can make patients feel the care and care of relatives, make the communication between patients and nursing staff closer, so as to overcome fear, reduce anxiety and depression, ensure peace of mind, and accept examination and treatment with a positive attitude. From this study, it is found that: The anxiety score and depression score of the observation group after nursing were lower than those of the control group (*P* < 0.05), and the examination time of the observation group was significantly shorter than that of the control group (*P* < 0.05). The comfort score and one-time success rate of the examination group were significantly higher than those of the control group (*P* < 0.05), the incidence of adverse reactions was significantly lower than that of the control group (*P* < 0.05), the excellent and good rate of image quality (95.00%) and nursing satisfaction (97.22%) were significantly higher than those of the control group (83.00%, 86.56%). This shows that the application effect of family care service mode in magnetic resonance enhanced scanning is remarkable, which can ensure the smooth development and completion of the examination, improve the patient's comfortable experience and improve the quality of nursing. This is mainly because the implementation of family care in MRI examination can avoid risk factors from many aspects. It can not only prevent the occurrence of adverse reactions and ensure the success of the examination, but also improve the patient's examination comfort and make the patient feel happy as much as possible.

## 5. Conclusion

The results of this study confirm that the implementation of family nursing service mode for patients undergoing MRI Dynamic enhancement scanning can effectively reduce the scores of anxiety and depression, shorten the examination time, reduce adverse reactions, improve the success rate of one-time examination, ensure the smooth development of MRI examination, improve the comfort of patients during examination and improve the scores of patients on nursing services. The effect is ideal and worthy of clinical research and promotion.

The article "Observation and Nursing of Adverse Reactions in Severe Patients with Enhanced MRI" was retracted in 2023. Reasons: suspected computer-generated content; unreliable results or conclusions; concerns about the data; concerns about the results or conclusions.

## Figures and Tables

**Figure 1:** Image reconstruction system and method technology in magnetic resonance imaging.

**Figure 2:** Comparison of inspection quality of two groups.

**Figure 3:** Comparison of nursing satisfaction between the two groups.

**Table 1:** Self rating Anxiety Scale (SAS)—standard.

Evaluation items	No or little	A small part of the time	Quite a lot of time	All time
1. I feel more nervous and anxious than usual				
2. I feel worried and scared for no reason				
3. I tend to get upset or panic				
4. I think I may be going crazy				
5. I feel that everything is going well and no bad luck will happen				
6. My limbs stir and tremble				
7. I am troubled by headache, neck pain and back pain				
8. I feel weak and tired easily				
9. I feel calm and can sit down quietly				
10. I Feel my heart beating fast				

**Table 2:** Evaluation of self rating Depression Scale (SDS).

Problem	No or very little	A small part of the time	Quite a lot of time	All time
1. I feel depressed and depressed				
2. I think the morning is the best of the day				
I Cry or want to cry				
4. I do not sleep well at night				
5. I eat as much as I used to				
6. I feel as happy as ever when I contact the opposite sex				
7. I find my weight is losing				
8. I have constipation				
9. My heart beats faster than usual				
10. I Feel tired for no reason				

**Table 3:** Comparison of anxiety and depression scores between the two groups$\left(\bar{x}\pm s\right)$

Group	Number of cases	Time	Anxiety score	Depression score
Control group	75	Before nursing	52.81 ± 5.42	51.62 ± 5.61
		After nursing	45.58 ± 3.16	45.14 ± 4.03
		T Value	6.513	5.576
		P	0.000	0.000

Observation group	75	Before nursing	52.53 ± 6.67	51.38 ± 5.54
		After nursing	41.47 ± 2.81	40.48 ± 3.56
		T Value	11.120	10.752
		P	0.000	0.000
		T1 value	0.155	0.110
		P	0.758	0.715
		T2 value	5.131	5.040
		P	0.000	0.000

*Note.* T1 and P1 are the comparison between groups before nursing; T2 and P2 are the comparison between the groups after nursing.

**Table 4:** Comparison of examination time and comfort scores between the two groups.$\left(\bar{x}\pm s\right)$

Group	Number of cases	Inspection time min	Comfort score
Control group	75	20.364.07	74.7810.45
Observation group	75	16.473.13	86.8312.06
T Value		6.366	-6.366
P		0.000	0.000

The article "Observation and Nursing of Adverse Reactions in Severe Patients with Enhanced MRI" was retracted in 2023. Reasons: suspected computer-generated content; unreliable results or conclusions; concerns about the data; concerns about the results or conclusions.

**Table 5:** Comparison of primary success rate and incidence of adverse reactions between the two groups.

Group	Number of cases	One time successful cases (%)	Dizzy	Adverse reactions (cases)			
				Nausea and vomiting	Skin flushing	Rash	Total occurrence
Control group	75	67(90.56)	4	2	3	1	12
Observation group	75	74(100.00)	2	0	1	0	3
X^2^ value		7.232	5.263				
P		<0.05					

**Table 6:** Comparison of image quality excellence rate.

Group	Number of cases	Excellent example	Good example	Poor example	Excellent rate%
Control group	75	26	35	11	83
Observation group	75	32	38	2	95

*Note.* The excellent and good rate of the two groups was 6.000, *P* < 0.05.

**Table 7:** Comparison of nursing satisfaction between the two groups.

Group	Number of cases	Very satisfied example	More satisfactory cases	Dissatisfaction example	Nursing satisfaction%
Control group	75	29	34	10	86.56
Observation group	75	33	38	1	97.22

*Note.* The comparison of satisfaction between the two groups, *x*^2^  = 5.797, *P* < 0.05.

## Data Availability

The datasets used and/or analyzed during the current study are available from the corresponding author on reasonable request.

## References

[1] Kim S.-H. (2020). Hydrogen Motion of CsH2PO4 Electrolyte Using 1H and 31P High-Resolution Nuclear Magnetic Resonance (NMR) Spectroscopy. *Science of Advanced Materials*.

[2] Carreo-Carrillo C. V., Sánchez E. V., Verduzco C. V., Herbert-Pucheta J. E. (2021). Polyphenol-based nuclear magnetic resonance non-targeted metabolomics of temperature- and time-controlled blue and red maize sprouting. *SN Applied Sciences*.

[3] Kozlowski A. M., Yates E. A., Roubroeks J. P., Tømmeraas K., Smith A. M., Morris G. A. (2021). Hydrolytic degradation of heparin in acidic environments: nuclear magnetic resonance reveals details of selective desulfation. *ACS Applied Materials & Interfaces*.

[4] Xu S., Zhu J., Zhao Q., Gao J., Zhang H., Hu B. (2021). Quality evaluation of cabernet sauvignon wines in different vintages by 1h nuclear magnetic resonance-based metabolomics. *Open Chemistry*.

[5] Witek M., Maciejaszek I., Surówka K. (2020). Impact of enrichment with egg constituents on water status in gluten-free rice pasta - nuclear magnetic resonance and thermogravimetric approach. *Food Chemistry*.

[6] Balthazar C. F., Guimarães J. T., Silva R. (2021). Effect of probiotic minas frescal cheese on the volatile compound and metabolic profiles assessed by nuclear magnetic resonance spectroscopy and chemometric tools. *Journal of Dairy Science*.

[7] Al Rashid K., Taylor A., Lumsden M. A., Goulding N., Lawlor D. A., Nelson S. M. (2020). Association of the serum metabolomic profile by nuclear magnetic resonance spectroscopy with sperm parameters: a cross-sectional study of 325 men. *F&S Science*.

The article "Observation and Nursing of Adverse Reactions in Severe Patients with Enhanced MRI" was retracted in 2023. Reasons: suspected computer-generated content; unreliable results or conclusions; concerns about the data; concerns about the results or conclusions.

[8] Masuda R., Kimura R., Karasaki T., Sase S., Goto K. (2021). Modeling the catalytic cycle of glutathione peroxidase by nuclear magnetic resonance spectroscopic analysis of selenocysteine selenenic acids. *Journal of the American Chemical Society*.

[9] Wang J., Dong S., Zhou C., Ashour A., Han B. (2021). Investigating pore structure of nano-engineered concrete with low-field nuclear magnetic resonance. *Journal of Materials Science*.

[10] Grunin Y. B., Grunin L. Y., Schiraya V. Y., Ivanova M. S., Masas D. S. (2020). Cellulose–water system’s state analysis by proton nuclear magnetic resonance and sorption measurements. *Bioresources and Bioprocessing*.

[11] Miao Y., Lam D., Zhuang J., Zhu J., Poget S. F., Tang M. (2020). Membrane topology of an ion channel detected by solid-state nuclear magnetic resonance and paramagnetic effects. *The Journal of Physical Chemistry Letters*.

[12] Wang J. Y., Guo Q. Y., Yao Z. Y. (2020). A low-field nuclear magnetic resonance dna-hydrogel nanoprobe for bisphenol a determination in drinking water. *Mikrochimica acta*.

[13] Wang S., Yang J., Shao G. (2020). Dilatational rheological and nuclear magnetic resonance characterization of oil-water interface: impact of ph on interaction of soy protein isolated and soy hull polysaccharides. *Food Hydrocolloids*.

[14] Reddy M. G., Lobo N. P., Ramanathan K. V., Narasimhaswamy T. (2020). Molecular Order of Topologically Variant Flexible Mesogens by 13C Nuclear Magnetic Resonance. *Langmuir*.

[15] Nawrocka E. K., Kasprzak P., Zawada K. (2019). Nonstationary two-dimensional nuclear magnetic resonance: a method for studying reaction mechanisms in situ. *Analytical Chemistry*.

[16] Huang X., Li A., Li X., Liu Y. (2019). Influence of typical core minerals on tight oil recovery during co_2 flooding using the nuclear magnetic resonance technique. *Energy & Fuels*.

[17] Jiang Y., Kwon K. D., Wang S., Ren C., Li W. (2019). Molecular speciation of phosphorus in phosphogypsum waste by solid-state nuclear magnetic resonance spectroscopy. *Science of The Total Environment*.

